The article "Knockdown of Long Non-Coding RNA KCNQ1OT1 Restrained Glioma Cells’ Malignancy by Activating miR-370/CCNE2 Axis" was retracted in 2023. Reason: concerns about the images.

# Knockdown of Long Non-Coding RNA KCNQ1OT1 Restrained Glioma Cells’ Malignancy by Activating miR-370/CCNE2 Axis

**DOI:** 10.3389/fncel.2017.00084

**Published:** 2017-03-22

**Authors:** Wei Gong, Jian Zheng, Xiaobai Liu, Yunhui Liu, Junqing Guo, Yana Gao, Wei Tao, Jiajia Chen, Zhiqing Li, Jun Ma, Yixue Xue

**Affiliations:** ^1^Department of Neurobiology, College of Basic Medicine, China Medical University Shenyang, China; ^2^Key Laboratory of Cell Biology, Ministry of Public Health of China, Key Laboratory of Medical Cell Biology, Ministry of Education of China, China Medical University Shenyang, China; ^3^Department of Neurosurgery, Shengjing Hospital of China Medical University Shenyang, China; ^4^Liaoning Research Center for Translational Medicine in Nervous System Disease Shenyang, China

**Keywords:** glioma, KCNQ1OT1, miR-370, CCNE2, hippo pathway

## Abstract

Accumulating evidence has highlighted the potential role of long non-coding RNAs (lncRNAs) as biomarkers and therapeutic targets in solid tumors. Here, we elucidated the function and possible molecular mechanisms of lncRNA KCNQ1OT1 in human glioma U87 and U251 cells. Quantitative Real-Time polymerase chain reaction (qRT-PCR) demonstrated that KCNQ1OT1 expression was up-regulated in glioma tissues and cells. Knockdown of KCNQ1OT1 exerted tumor-suppressive function in glioma cells. Moreover, a binding region was confirmed between KCNQ1OT1 and miR-370 by dual-luciferase assays. qRT-PCR showed that miR-370 was down-regulated in human glioma tissue and cells. In addition, restoration of miR-370 exerted tumor-suppressive function via inhibiting cell proliferation, migration and invasion, while promoting the apoptosis of human glioma cells. Knockdown of KCNQ1OT1 decreased the expression level of Cyclin E2 (CCNE2) by binding to miR-370. Further, miR-370 bound to CCNE2 3′UTR region and decreased the expression of CCNE2. These results provided a comprehensive analysis of KCNQ1OT1-miR-370-CCNE2 axis in human glioma cells and might provide a novel strategy for glioma treatment.

## Introduction

Gliomas are one of the most life-threatening and common primary human brain malignancies with an annual incidence of five cases per 100,000 people. Despite advancements in surgery and adjuvant therapy, the prognosis remains very poor, with a median survival of less than 15 months (Xu et al., 2010; Li et al., 2014).

Long non-coding RNAs (lncRNAs) have been confirmed to act as key molecules in cancer development and progression (Cloutier et al., 2016; Liu et al., 2016). Dysregulations of lncRNAs are discovered in various tumor tissues and cancer cells where they serve as oncogenes or tumor suppressors (Ellinger et al., 2015; Jiang et al., 2016). KCNQ1OT1, an imprinted antisense lncRNA in the human KCNQ1 locus on chromosome 11p15.5, is involved in cis-limited silencing within an imprinted KCNQ1 cluster (Zhang et al., 2014; Sunamura et al., 2016). Earlier studies showed that KCNQ1OT1 was up-regulated in breast cancer and conferred to breast cancer malignancy (Zhang et al., 2016a). Similarly, over-expressed KCNQ1OT1 contributed to the carcinogenesis of hepatocellular carcinoma (Wan et al., 2013). However, the expression and function of KCNQ1OT1 in glioma remain unclear.

The article "Knockdown of Long Non-Coding RNA KCNQ1OT1 Restrained Glioma Cells’ Malignancy by Activating miR-370/CCNE2 Axis" was retracted in 2023. Reason: concerns about the images.

MicroRNAs (miRNAs) play crucial roles in post-transcriptional gene regulation and serve as negative gene regulators by targeting 3′-UTR of downstream genes (Karsy et al., 2012). MiRNAs have emerged as key regulators in cancer cell biology including cell proliferation, migration, invasion and apoptosis (Zhao et al., 2015). Aberrant expression of miR-370 has been reported in various cancers. In most cases, miR-370 serves as a tumor-suppressive gene in tumors such as liver cancer and osteosarcoma (Duan et al., 2015; Sun G. et al., 2016). More importantly, miR-370 has been confirmed to be down-regulated in glioma and reduces glioma cells growth (Peng et al., 2016). But the detailed function of miR-370 still needs to be explored.

Cyclin E2 (CCNE2) is a member of cyclin E family, and one of its major function is making transition from G0/G1 to S phase through binding with CDK2 and phosphorylation of Rb protein (Bizama et al., 2014; Ng et al., 2014; Cong et al., 2015). CCNE2 expression was found to be dysregulated in many cancers such as breast cancer and thyroid cancer (Payton et al., 2002; Liang et al., 2015). However, the characterization of CCNE2 in glioma has not been investigated.

In the present study, we investigated the expression and function of KCNQ1OT1, miR-370 and CCNE2 in glioma tissues and cells. We also studied the underlying interactions among them. There was a specific binding site between KCNQ1OT1 and miR-370. KCNQ1OT1 and miR-370 negatively regulated their respective expression. MiR-370 targeted CCNE2 3′-UTR and impaired its expression. We hypothesized KCNQ1OT1/miR-370/CCNE2 might exert crucial function in glioma cells progression and might be a novel therapeutic target.

## Materials and Methods

### Clinical Tumors

All human glioma tumors and normal brain tumors (NBTs) were collected from the Department of Neurosurgery, Shengjing Hospital of China Medical University, from 2013 to 2016. Glioma samples were divided into four groups: Grade I, Grade II, Grade III and Grade IV, according to the World Health Organization (WHO) classification. Informed consent was obtained from all patients and the study procedure was approved by Research Ethics Board at the Shengjing Hospital of China Medical University. The tumor specimens were immediately frozen and preserved in liquid nitrogen until used in our research.

The article "Knockdown of Long Non-Coding RNA KCNQ1OT1 Restrained Glioma Cells’ Malignancy by Activating miR-370/CCNE2 Axis" was retracted in 2023. Reason: concerns about the images.

### Cell Culture

Human glioma cell lines (U87, U251) and human embryonic kidney (HEK) 293T cells were acquired from Shanghai Institutes for Biological Sciences Cell Resource Center. They were cultured in high glucose Dulbecco’s Modified Eagle Medium (DMEM) supplemented with 10% fetal bovine serum (FBS, Gibco, Carlsbad, CA, USA). Primary normal human astrocytes (NHA) were obtained from Sciencell Research Laboratories (Carlsbad, CA, USA) and cultured in astrocyte medium (Carlsbad, CA, USA). All cells were incubated at 37°C a humidified incubator with 5% CO_2_.

### RNA Extraction and Quantitative Real-Time PCR (qRT-PCR)

We used trizol reagent (Life Technologies Corporation, Carlsbad, CA, USA ) extracted total RNA from NBTs, glioma tissues, NHA, U87 and U251 cell lines. The primers for KCNQ1OT1 and GAPDH were synthesized from Takara Bio (Japan). The primers for miR-370 and U6 were synthesized from the Applied Biosystems. RNA concentration and quality were measured by the 260/280 nm ratio using a Nanodrop Spectrophotometer (ND-100, and we used One-Step SYBR PrimeScript RT-PCR Kit (Perfect Real Time; Takara Bio, Inc., Japan) to test the expression of KCNQ1OT1 in NBTs, glioma tissues, NHA, U87 and U251 cells. KCNQ1OT1: forward 5′-TGCAGAAGACAGGACACTGG-3′, reverse 5′-CTTTGGTGGGAAAGGACAGA-3′; GAPDH: forward 5′-TGCACCACCAACTGCTTAGC-3′, reverse 5′-GGCATGCACTGTGGTCATGAG-3′. GAPDH was used as endogenous controls for genes expressions. High Capacity cDNA Reverse Transcription Kits (Applied Biosystems, Foster City, CA, USA) and Taqman Universal Master Mix II (Life Technologies Corporation, Carlsbad, CA, USA) were used to examine the expression levels of miR-370 and U6 (Applied Biosystems, Foster City, CA, USA) levels. Fold change was calculated as 2^−∆∆Ct^ in gene expression.

### Cell Transfections

Short-hairpin KCNQ1OT1 (sh-KCNQ1OT1) plasmid and its respective non-targeting sequence (negative control, sh-NC), miR-370 agomir (pre-miR-370), miR-370 antagomir (anti-miR-370) and their respective non-targeting sequence (negative control, NC; pre-NC or anti-NC) were synthesized as previously described (GenePharma, Shanghai, China; Zhou et al., 2009; Wang and Li, 2010; Wang et al., 2012). CCNE2 full length (with 3′UTR) plasmid, CCNE2 (without 3′UTR) plasmid and their respective non-targeting sequence (negative control, NC) were synthesized as previously described (Life technology, Waltham, MA, USA; Pleet et al., 2016). We used Opti-MEM and Lipofectamine 3000 reagent (Life Technologies Corporation, Carlsbad, CA, USA) for transfection when cells were at 50%–70% confluence. Stable cell lines were obtained through the selection by means of Geneticin (G418; Sigma-Aldrich, St. Louis, MO, USA), G418-resistant clones were obtained after 3–4 weeks. We used qRT-PCR to detect the knockdown efficiency.

The article "Knockdown of Long Non-Coding RNA KCNQ1OT1 Restrained Glioma Cells’ Malignancy by Activating miR-370/CCNE2 Axis" was retracted in 2023. Reason: concerns about the images.

### Cell Proliferation Assay

After knockdown efficacy was confirmed, cell counting Kit-8 (CCK-8, Dojin, Japan) assay was used for cell proliferation. Two-thousand cells were seeded per well in 96-well plates at a same density, and 10 μL of Cell Counting Kit-8 was added into each well after 48 h. Then incubated at 37°C for 2 h and absorbance was measured at 450 nm.

### Apoptosis Detection

Apoptosis was evaluated using Annexin V-PE/7-AAD staining apoptosis detection kit (Southern Biotech, Birmingham, AL, USA) according to the manufacturer’s instructions. After the cells washed two times with 4°C PBS, cells were collected and stained with Annexin V-PE and 7-AAD. Then acquired the cells by flow cytometry (FACScan, BD Biosciences, San Jose, CA, USA) and analyzed by CELL Quest 3.0 software.

### Cell Migration and Invasion Assay

The abilities of cell migration and invasion were tested using the 24-well transwell chambers with 8 μm pore size polycarbonate membrane (Corning, NY, USA). For cell invasion assay, the filter was pre-coated with 500 ng/ml matrigel solution (BD, Franklin Lakes, NJ, USA) and incubated at 37°C for 4 h before the invasion assay started; placed 500 μL of 10% FBS medium in the lower chamber, and placed 100 μL serum-free medium in the upper chamber. After incubation at 37°C for 24 h, the cells on the upper membrane surface were scraped off. Surface were fixed with methanol and glacial acetic acid 30 min and then stained with 10% Giemsa solution. Number of cells was counted, and five randomly fields were counted randomly in each well. The photographs were taken at 200× magnification.

### Luciferase Reporter Assays

KCNQ1OT1 full length and CCNE2 3′-UTR sequences were amplified by PCR and cloned into a pmirGlo Dual-luciferase miRNA Target Expression Vector (Promega, Madison, WI, USA) to construct luciferase reporter vector (KCNQ1OT-Wt and CCNE2-Wt; GenePharma). The sequence of putative binding site was replaced as indicated (KCNQ1OT1-Mut and CCNE2-Mut) to mutate the putative binding sites of KCNQ1OT1 or CCNE2. HEK-293T cells were seeded in 96-well plates and the cells were co-transfected with KCNQ1OT1-Wt (or KCNQ1OT1-Mut) or CCNE2-Wt (or CCNE2-Mut) and miR-370 or miR-370-NC plasmids when they reached 50%–70% confluence. The luciferase activities were measured at 48 h after transfection by Dual-Luciferase reporter assay kit (Promega). The cells were divided in five groups respectively: control group, KCNQ1OT1-Wt + miR-370-NC (transfected with KCNQ1OT1-Wt and pre-NC), KCNQ1OT1-Wt + miR-370 group (transfected with KCNQ1OT1-Wt and pre-miR-370), KCNQ1OT1-Mut + miR-370-NC group (transfected with KCNQ1OT1-Mut and pre-NC), KCNQ1OT1-Mut + miR-370 group (transfected with KCNQ1OT1-Mut and pre-miR-370); Control group, CCNE2-Wt + miR-370-NC (transfected with CCNE2-Wt and pre-NC), CCNE2-Wt + miR-370 group (transfected with CCNE2-Wt and pre-miR-370), CCNE2-Mut + miR-370-NC group (transfected with CCNE2-Mut and pre-NC), CCNE2-Mut + miR-370 group (transfected with CCNE2-Mut and pre-miR-370).

The article "Knockdown of Long Non-Coding RNA KCNQ1OT1 Restrained Glioma Cells’ Malignancy by Activating miR-370/CCNE2 Axis" was retracted in 2023. Reason: concerns about the images.

### RNA Immunoprecipitation

RNA immunoprecipitation was performed as previously reported (Zheng et al., 2016). Briefly, to explore whether KCNQ1OT1 and miR-370 were associated with the RISC, we performed RNA immunoprecipitation. Glioma cells were lysed in complete RNA lysis buffer with protease inhibitor and RNase inhibitor from an EZ-Magna RIP RNA-binding protein immunoprecipitation kit (Millipore, Billerica, MA, USA). Whole cell lysates from the control groups and miR-370 groups were incubated with RIP immunoprecipitation buffer containing magnetic beads conjugated with human anti-Argonaute 2 antibody (Millipore, Billerica, MA, USA) and the negative control (normal mouse IgG; Millipore, Billerica, MA, USA). Samples were incubated with Proteinase K buffer, and then the immunoprecipitated RNA was isolated. Purified RNA was obtained and qRT-PCR was performed with the primers mentioned above to illustrate the presence of the binding targets.

### Western Blot Analysis

Total protein of cells were lysed using ice-cold RIPA (Beyotime Institute of Biotechnology) buffer supplemented with protease inhibitors and centrifuged at 17,000× g 4°C for 40 min. Equal amount of total cell lysate protein samples (40 μg) went electrophoresis in sodium dodecyl sulfate-polyacrylamide gel electrophoresis (SDS-PAGE) and then Equal amount of total cell lysate protein samples (40 μg) went electrophoresis in SDS-PAGE and then transferred to polyvinylidene difluoride membranes. Membranes were incubated in 5% nonfat milk dissolved in Tris-buffered saline (TBS) containing 0.1% Tween-20 for 2 h at room temperature. After blocking of non-specific bindings, the protein went immunoblotting with primary antibodies against CCNE2 (1:200, Santa Cruz Biotechnology, Santa Cruz, CA, USA), YAP1 (1:1000, Santa Cruz Biotechnology, Santa Cruz, CA, USA), p-YAP (1:2000, CST, USA) and GAPDH (1:1000, Proteintech, Chicago, IL, USA). Followed by incubation with appropriate correlated HRP-conjugated secondary antibody, then the membranes were incubated with secondary antibodies (goat anti-rabbit or goat anti-mouse, 1:5000 respectively; Santa Cruz Biotechnology, Santa Cruz, CA, USA) at room temperature for 2 h. Immunoblots were visualized by enhanced chemiluminescence (ECL kit, Santa Cruz Biotechnology, Santa Cruz, CA, USA) and scanned using ChemImager 5500 V2.03 software. The integrated density values (IDV) were calculated using FluorChem 2.0 software.

The article "Knockdown of Long Non-Coding RNA KCNQ1OT1 Restrained Glioma Cells’ Malignancy by Activating miR-370/CCNE2 Axis" was retracted in 2023. Reason: concerns about the images.

### Subcutaneous and Orthotopic Xenografts in Nude Mice

The stably transfected human glioma tissues were used in the *in vivo* study. Four-week-old male nude mice were purchased from the National Laboratory Animal Center (Beijing, China). All mice were free to autoclaved food and water during the experiment, and all experiments with nude mice were performed strictly in accordance with a protocol approved by the Administrative Panel on Laboratory Animal Care of the China Medical University. Lentivirus encoding miR-370 was generated using pLenti6.3/V5eDEST Gateway Vector Kit (Life Technologies Corporation, Carlsbad, CA, USA). The miR-370 and short-hairpin RNA targeting human KCNQ1OT1 were ligated into the pLenti6.3/V5eDEST vector and LV3-CMV-GFP-Puro vector (GenePharma, Shanghai, China), respectively, and then pLenti6.3/V5eDEST-miR-370 and LV3-CMV-GFPPuro-sh-KCNQ1OT1 vectors were generated. The ViraPower Packaging Mix was used to generate Lentivirus in 293FT cells. After infection, the stable expressing cells of miR-370 and sh-KCNQ1OT1 were obtained. The lentiviruses of miR-370 were transduced in sh-KCNQ1OT1 stably transfected cells to generate miR-370 + sh-KCNQ1OT1 cells. The nude mice were divided into four groups: control group (only U87 or U251), sh-KCNQ1OT1 group (sh-KCNQ1OT1 stable expression U87 or U251 cells), miR-370 group (miR-370 stable over-expression U87 or U251 cells) and sh-KCNQ1OT1 + miR-370 group (KCNQ1OT1 inhibition and miR-370 over-expression stable U87 and U251 cells). 3 × 10^5^ cells were subcutaneously injected in the right flanks of the mice. Tumor volume was measured every 4 days when the tumors were obviously identified and the volume was calculated by the formula: volume (mm^3^) = length × width^2^/2. Fourty-four days after injection, mice were sacrificed and tumors were isolated. As previously described (Rubin et al., 2003; Zhou et al., 2015), for survival analysis in orthotopic inoculations, 3 × 10^5^ cells were stereotactically implanted into the right striatum of the mice in the position of 2 mm posterior to the bregma, 2 mm laterally, and 2 mm deep to the dura. The number of survived nude mice was marked and survival analysis was investigated using Kaplane-Meier survival curve.

The article "Knockdown of Long Non-Coding RNA KCNQ1OT1 Restrained Glioma Cells’ Malignancy by Activating miR-370/CCNE2 Axis" was retracted in 2023. Reason: concerns about the images.

### Statistical Analysis

Data are presented as mean ± standard deviation (SD). SPSS 18.0 statistical software with the Student’s *t*-test or one-way analysis of variance (ANOVA) were used to evaluate all statistical analyses. Multiple comparison between the groups was performed using S-N-K method. Differences were considered to be significant when *P* < 0.05.

## Results

### KCNQ1OT1 was Up-Regulated in Glioma Tissues and Cell Lines, KCNQ1OT1 Inhibition Impeded Glioma Cells Malignant Progression

The latest studies confirmed aberrant KCNQ1OT1 expression was ubiquitous in various tumors. We first investigated KCNQ1OT1 expression in glioma tissues and cells. As Figures 1A,B showed, the expression of KCNQ1OT1 in glioma tissues and cell lines was robustly up-regulated in glioma tissues (*P* < 0.01), U87 and U251 cells (*P* < 0.05), and was positively correlated with the histopathological grades of gliomas. Therefore, we hypothesized KCNQ1OT1 might contribute to glioma cells’ malignancy. U87 and U251 cells with stable inhibition of KCNQ1OT1 were established. We then examined the knockdown efficiency (Figure 1C; *P* < 0.01). As expected, cell proliferation was reduced in sh-KCNQ1OT1 group compared with sh-NC group (Figure 1D; *P* < 0.05). Similarly, flow cytometry results showed that down-regulation of KCNO1OT1 induced glioma cells apoptosis compared with sh-NC group (Figure 1E; *P* < 0.05). Further, as shown in Figure 1F, U87 and U251 cells’ migration and invasion ability were weaker in experiment group compared with sh-NC group (*P* < 0.05). These results indicate KCNQ1OT1 acts as an oncogene in glioma cells.

**Figure 1:** **KCNQ1OT1 expression in glioma tissues and human glioma cells**. Knockdown of KCNQ1OT1 restrained cell proliferation, promoted apoptosis and restrained migration and invasion in human glioma cells. **(A)** KCNQ1OT1 expression in normal brain tissues (NBTs), different grades of human glioma tissues. Data are presented as the mean ± standard deviation (SD; *n* = 15, each group). *P < 0.01 vs. NBTs group. **(B)** Expression levels of KCNQ1OT1 in human normal astrocytes and human glioma cell lines U87 and U251. Data are presented as the mean ± SD (*n* = 5, each group). *P < 0.01 vs. Normal human astrocytes (NHA) group. **(C)** Knockdown efficiency of KCNQ1OT1 inhibition. **(D)** CCK-8 assay was used to determine the proliferation effect of KCNQ1OT1 on human glioma cells. **(E)** Flow cytometry analysis of KCNQ1OT1 knockdown on glioma cells. **(F)** Quantification of migration and invasion of KCNQ1OT1 knockdown of human glioma cells. Representative images and accompanying statistical plots were presented. Data are presented as the mean ± SD (*n* = 5, each group). *P < 0.05 vs. sh-NC group. Scale bars represent 20 μm. **P < 0.01 vs. NBTs group.

The article "Knockdown of Long Non-Coding RNA KCNQ1OT1 Restrained Glioma Cells’ Malignancy by Activating miR-370/CCNE2 Axis" was retracted in 2023. Reason: concerns about the images.

### Over-Expression of miR-370 Impaired Cell Proliferation, Migration and Invasion, While Promoted Apoptosis of Glioma Cells

An earlier study has shown miR-370 was down-regulated in glioma tissues and cells (Peng et al., 2016). In addition, the restoration of miR-370 reduced glioma cells proliferation. We further explored miR-370’s detailed function in glioma cells. Consistent with previously reported, CCK-8 assay indicated over-expression of miR-370 restrained the proliferation of U87 and U251 cells compared with pre-NC group at different times (Figure 2A; *P* < 0.05). Meanwhile, over-expression of miR-370 led to an increased ratio in apoptosis compared with pre-NC group (Figure 2B; *P* < 0.05). Transwell assays were conducted to assess the effects of miR-370 on the migratory and invasive abilities of glioma cells. As Figure 2C showed, the number of cells was reduced in pre-miR-370 group compared with pre-NC group (*P* < 0.05). Therefore miR-370 might act as a tumor suppressor in glioma cells.

**Figure 2:** **Effect of miR-370 on proliferation, migration, invasion and apoptosis of human glioma cells. (A)** Cell counting Kit-8 (CCK-8) assay was used to determine the proliferation effect of miR-370 on human glioma cells at 24 h, 48 h and 72 h. **(B)** Flow cytometry analysis of human glioma cells with the expression of miR-370 changed. **(C)** Quantification of migration and invasion cells with the expression of miR-370 changed. Representative images and accompanying statistical plots were presented. Data are presented as the mean ± SD (*n* = 5, each group). *P < 0.05 vs. pre-NC group; ^#^*P* < 0.05 vs. anti-NC group. Scale bars represent 20 μm.

### MiR-370 Mediated the Tumor-Suppressive Effect of KCNQ1OT1’s Inhibition on Glioma Cells

Multiple studies have confirmed lncRNAs harbor miRNAs binding sites (Su et al., 2016). LncRNAs can sponge miRNAs in a sequence-specific manner (Ballantyne et al., 2016). In most cases, lncRNAs and miRNAs regulate expression respectively in an Argonaute2-dependent manner (Kobayashi and Tomari, 2016). We used a bioinformatics database (Starbase) to infer the potential targets of miR-370. KCNQ1OT1 was identified as a potential target and harbored one putative binding site of miR-370. We first examined the expression of miR-370 in KCNQ1OT1 inhibition glioma cells. As shown in Figure 3A, miR-370 expression was increased in sh-KCNQ1OT1 group compared with sh-NC group (*P* < 0.01). Further, as shown in Figure 3A, we found KCNQ1OT1 expression was negatively correlated with miR-370 expression in glioma cells (*P* < 0.01). Luciferase assays were used to confirm the functional binding site between KCNQ1OT1 and miR-370. The binding site and the designed mutated site are shown in Figure 3B. As shown in Figure 3C, luciferase activity was significantly reduced in KCNQ1OT1-WT + miR-370 group compared with KCNQ1OT1-WT + miR-370-NC group (*P* < 0.05). We further performed RNA-binding protein immunoprecipitation (RIP) experiment to ascertain whether KCNQ1OT1 and miR-370 were in a RNA-induced silencing complex (RISC). As shown in Figure 3D, KCNQ1OT1 and miR-370 were both detected in anti-Ago2 group (*P* < 0.01). These results demonstrated an insight into the mechanism of KCNQ1OT1 negatively regulating miR-370.

The article "Knockdown of Long Non-Coding RNA KCNQ1OT1 Restrained Glioma Cells’ Malignancy by Activating miR-370/CCNE2 Axis" was retracted in 2023. Reason: concerns about the images.

**Figure 3:** **MiR-370 targeted KCNQ1OT1 and its expression was negatively correlative with KCNQ1OT1, miR-370 was involved in KCNQ1OT1-mediated regulation of human glioma cells. (A)** Quantitative Real-Time polymerase chain reaction (qRT-PCR) analysis for miR-370 expression negatively correlative with KCNQ1OT1 in human glioma cell lines. Data are presented as the mean ± SD (*n* = 5, each group). **P < 0.01 vs. sh-NC group. **P < 0.01 vs. pre-NC; ^##^*P* < 0.01 vs. sh-NC group. **(B)** KCNQ1OT1 harbored a putative miR-370 binding site, and designed mutant sequences were indicated. **(C)** Dual-luciferase reporter assay of human embryonic kidney (HEK) 293T cells co-transfected with KCNQ1OT1-WT and miR-370-NC or KCNQ1OT1-WT and miR-370, and KCNQ1OT1-Mut and miR-370-NC or KCNQ1OT1-Mut and miR-370. Data are presented as the mean ± SD (*n* = 5, each group). *P < 0.05 vs. KCNQ1OT1-WT + miR-370-NC group. **(D)** MiR-370 was identified in KCNQ1OT1-RISC complex. KCNQ1OT1 and miR-370 expression levels were measured using qRT-PCR (Data represent mean ± SD (*n* = 5, each group). ^&&^*P* < 0.01 vs. anti-normal IgG group. **(E)** CCK-8 assay was used to evaluate the effect of KCNQ1OT1 and miR-370 on cell proliferation in human glioma cells at 24 h, 48 h and 72 h. Data are presented as the mean ± SD (*n* = 5, each group). *P < 0.05 vs. sh-NC + pre-NC group. **(F)** Flow cytometry analysis was used to evaluate the effect of KCNQ1OT1 and miR-370 on cell apoptosis in human glioma cells. Data are presented as the mean ± SD (*n* = 5, each group). *P < 0.05 vs. sh-NC + pre-NC group. **(G)** Quantification of cells to evaluate the effect of KCNQ1OT1 and miR-370 on cell migration and invasion in human glioma cells. Data are presented as the mean ± SD (*n* = 5, each group). *P < 0.05 vs. sh-NC + pre-NC group. Scale bars represent 20 μm.

To determine whether miR-370 conferred to the tumor-suppressive effect of KCNQ1OT1’s inhibition, we transfected over-expression of miR-370 or miR-370 inhibitors into the stable sh-KCNQ1OT1 cells prior to the assessment of cell proliferation, apoptosis, migration and invasion. As shown in Figure 3E, sh-KCNQ1OT1 cells co-transfected with over-expression of miR-370 had the strongest inhibitory effect on cell proliferation compared with sh-NC + pre-NC group at different times (*P* < 0.05). Flow cytometry results showed that glioma cells treated with sh-KCNQ1OT1 + pre-miR-370 exhibited increased apoptotic ratio compared with sh-NC + pre-NC group (Figure 3F; *P* < 0.05). Similarly, knockdown of KCNQ1OT1 combined with restoration of miR-370 robustly decreased migrating and invading glioma cells (Figure 3G; *P* < 0.05).

The article "Knockdown of Long Non-Coding RNA KCNQ1OT1 Restrained Glioma Cells’ Malignancy by Activating miR-370/CCNE2 Axis" was retracted in 2023. Reason: concerns about the images.

### CCNE2 was Involved in KCNQ1OT1/miR-370-Mediated Glioma Cells Malignant Progression

CCNE2 exerts oncogenetic function in various tumors such as breast cancer and bladder cancer (Gupta et al., 2016). We first detected the expression of CCNE2 in glioma tissues using western blot. As shown in Figure 4A, CCNE2 expression were obviously up-regulated in high- and low-grade glioma tissues compared with normal brain tissues (NBTs; *P* < 0.05). CCNE2 was identified as one of the downstream genes of miR-370 by Bioinformatics database (Targetscan, miRanda and Starbase). Luciferase reporter assay was performed to verify the putative binding site between miR-370 and CCNE2. The binding site and the designed mutated site are shown in Figure 4B. As shown in Figure 4C, luciferase activity was significantly reduced in CCNE2-Wt + miR-370 group compared with CCNE2-Wt + miR-370-NC group (*P* < 0.05).

**Figure 4:** **Cyclin E2 (CCNE2) was up-regulated in glioma tissues**. CCNE2 was a target of miR-370, both KCNQ1OT1 and miR-370 could modulate CCNE2 expression. **(A)** CCNE2 protein expression levels in normal brain tissues and glioma tissues using GAPDH as an endogenous control. Representative protein expression and their integrated light density values (IDVs) of CCNE2 in normal brain tissues, low-grade glioma tissues ([WHO] I-II), and high-grade glioma tissues ([WHO] III-IV) are shown. Data are presented as the mean ± SD (*n* = 5, each group). *P < 0.05 vs. NBTs group. **(B)** CCNE2 harbored a putative miR-370 binding site, and designed mutant sequences were indicated. **(C)** Dual-luciferase reporter assay of HEK 293T cells co-transfected with CCNE2-Wt and miR-370-NC or CCNE2-Wt and miR-370, and CCNE2-Mut and miR-370-NC or CCNE2-Mut and miR-370. Data are presented as the mean ± SD (*n* = 5, each group). *P < 0.05 vs. CCNE2-Wt + miR-370-NC group. **(D)** Western blot analysis for CCNE2 in KCNQ1OT1 knockdown of human glioma cells using GAPDH as an endogenous control. Data are presented as the mean ± SD (*n* = 5, each group). *P < 0.05 vs. sh-NC group. **(E)** Western blot analysis for CCNE2 in miR-370 over-expression and miR-370 inhibition of human glioma cells using GAPDH as an endogenous control. Data are presented as the mean ± SD (*n* = 5, each group). *P < 0.05 vs. pre-NC group; ^#^*P* < 0.05 vs. anti-NC group. **(F)** Western blot analysis for CCNE2 in co-transfected KCNQ1OT1 inhibition with miR-370 over-expression or miR-370 inhibition of human glioma cells using GAPDH as an endogenous control. Data are presented as the mean ± SD (*n* = 5, each group). *P < 0.05 vs. sh-NC + pre-NC group.

The article "Knockdown of Long Non-Coding RNA KCNQ1OT1 Restrained Glioma Cells’ Malignancy by Activating miR-370/CCNE2 Axis" was retracted in 2023. Reason: concerns about the images.

Further, we examined the expression of CCNE2 protein in cells treated with KCNQ1OT1 or miR-370. As shown in Figure 4D, CCNE2 protein level was decreased in sh-KCNQ1OT1 group compared with sh-NC group (*P* < 0.05). CCNE2 protein levels were also examined in overexpressed or inhibited miR-370 cells. As expected, CCNE2 protein level was attenuated in pre-miR-370 group, while it was up-regulated in anti-miR-370 group (Figure 4E; *P* < 0.05). Having confirmed both KCNQ1OT1 and miR-370 affected glioma cells’ malignant biological behaviors, we further investigated the underlying molecular mechanisms. Figure 4F showed that CCNE2 protein expression was robustly decreased in sh-KCNQ1OT1 + pre-miR-370 group, while anti-miR-370 rescued sh-KCNQ1OT1 induced down-regulation of CCNE2 protein expression (*P* < 0.05).

### CCNE2 Promoted Cell Proliferation, Migration and Invasion, While Inhibited Apoptosis of Glioma Cells

Having confirmed CCNE2 was up-regulated in glioma cells and participated in KCNQ1OT1/miR-370 regulating glioma cells’ malignancy, we examined the effect of CCNE2 on glioma cells’ biological behaviors. CCK-8 assay indicated over-expression of CCNE2 (CCNE2 (+)) promoted the proliferation of glioma U87 and U251 cells compared with CCNE2 (+)-NC group (Figure 5A; *P* < 0.05). Meanwhile, over-expression of CCNE2 (CCNE2 (+)) led to a decreased apoptotic ratio of glioma cells compared with CCNE2 (+)-NC group (Figure 5B; *P* < 0.05). Transwell assays were conducted to assess the effects of CCNE2 (+) on the migratory and invasive ability of glioma cells. As expected, the migratory and invasive ability was stronger in CCNE2 (+) group compared with CCNE2 (+)-NC group (Figure 5C; *P* < 0.05).

**Figure 5:** **Effect of CCNE2 on proliferation, migration, invasion and apoptosis of human glioma cells. (A)** CCK-8 assay was used to determine the proliferation effect of CCNE2 on human glioma cells. *P < 0.05 vs. CCNE2 (+)-NC group; ^#^*P* < 0.05 vs. CCNE2 (−)-NC group. **(B)** Flow cytometry analysis of human glioma cells with the expression of CCNE2 changed. *P < 0.05 vs. CCNE2 (+)-NC group; ^#^*P* < 0.05 vs. CCNE2 (−)-NC group. **(C)** Quantification of migration and invasion cells with the expression of CCNE2 changed. Representative images and accompanying statistical plots were presented. *P < 0.05 vs. CCNE2 (+)-NC group; ^#^*P* < 0.05 vs. CCNE2 (−)-NC group. Scale bars represent 20 μm.

The article "Knockdown of Long Non-Coding RNA KCNQ1OT1 Restrained Glioma Cells’ Malignancy by Activating miR-370/CCNE2 Axis" was retracted in 2023. Reason: concerns about the images.

### CCNE2 Reversed KCNQ1OT1 Knockdown Phenotype

To investigate whether over-expression of CCNE2 reversed KCNQ1OT1 knockdown phenotype, cells expressed sh-KCNQ1OT1 + CCNE2 were established. CCK-8 assay showed that over-expression of CCNE2 reversed inhibitory of proliferation sh-KCNQ1OT1 induced (Figure 6A; *P* < 0.05). Further, over-expression of CCNE2 rescued increased apoptotic ratio sh-KCNQ1OT1 induced of glioma cells (Figure 6B; *P* < 0.05). Meanwhile, Figure 6C showed that over-expression of CCNE2 reversed inhibitory of migratory and invasive ability sh-KCNQ1OT1 induced of glioma cells.

**Figure 6:** **Sh-KCNQ1OT1 phenotype was reversed by over expression of CCNE2. (A)** CCK-8 assay was used to determine the proliferation effect of sh-KCNQ1OT1 + CCNE2 on human glioma cells. *P < 0.05 vs. Control group; ^#^*P* < 0.05 vs. sh-KCNQ1OT1 group. **(B)** Flow cytometry analysis of human glioma cells with the expression of CCNE2 changed. *P < 0.05 vs. Control group; ^#^*P* < 0.05 vs. sh-KCNQ1OT1 group. **(C)** Quantification of migration and invasion cells with the expression of CCNE2 changed. Representative images and accompanying statistical plots were presented. *P < 0.05 vs. Control group; ^#^*P* < 0.05 vs. sh-KCNQ1OT1 group. Scale bars represent 20 μm.

### Reintroduction of miR-370 Impaired CCNE2-Induced Promotion Effects on Glioma U87 and U251 Cells by Targeting CCNE2 3′-UTR

To discover whether CCNE2 reversed miR-370-mediated blocking of glioma U87 and U251 cells’ malignant evolution in a sequence-specific manner, we analyzed proliferation, migration, invasion and apoptosis of U87 and U251 which stably expressed miR-370 + CCNE2 (non-3′UTR). The proliferation of glioma cells in miR-370 + CCNE2 (non-3′UTR) group was significantly rescued compared with miR-370 + CCNE2 group at different times (Figure 7A; *P* < 0.05). Cells treated with miR-370 + CCNE2 (non-3′UTR) exhibited a vigorously reduced apoptotic ratio in U87 and U251 cells compared with miR-370 + CCNE2 group (Figure 7B; *P* < 0.05). Moreover, Figure 7C showed that the number of migrating and invading cells were increased in miR-370 + CCNE2 (non-3′UTR) group compared with miR-370 + CCNE2 group (*P* < 0.05).

**Figure 7:** **MiR-370 inhibited human glioma cells malignant progression via targeting to CCNE2 3′-UTR**. CCNE2 activated the YAP1 signal pathways. **(A)** CCK-8 assay was used to evaluate the proliferation effect of miR-370 and CCNE2 changed on human glioma cells at 24 h, 48 h and 72 h. **(B)** Flow cytometry analysis of human glioma cells with the expression of miR-370 and CCNE2 changed. **(C)** Quantification of migration and invasion cells with the expression of miR-370 and CCNE2 changed. Representative images and accompanying statistical plots were presented. Data are presented as the mean ± SD (*n* = 5, each group). *^#^*P* < 0.05 vs. miR-370 + CCNE2 group. Scale bars represent 20 μm. **(D)** Western blot analysis of the YES-associated protein (YAP) pathways regulated by CCNE2 in human glioma cells. Data are presented as the mean ± SD (*n* = 5, each group). *^▲^^#^*P* < 0.05 vs. Sh-KCNQ1OT1 group and pre-miR-370 group.

The article "Knockdown of Long Non-Coding RNA KCNQ1OT1 Restrained Glioma Cells’ Malignancy by Activating miR-370/CCNE2 Axis" was retracted in 2023. Reason: concerns about the images.

A latest study showed CCNE2 promoted breast cancer cells’ malignant progression via activating Hippo pathway (Pegoraro et al., 2015). Therefore, we detected p-YAP and YES-associated protein (YAP) expression in cells treated with KCNQ1OT1 and miR-370. As shown in Figure 7D, p-YAP expression was up-regulated in sh-KCNQ1OT1 group and pre-miR-370 group compared with control group (*P* < 0.05). Besides, p-YAP expression was robustly increased in sh-KCNQ1OT1 + pre-miR-370 group.

### KCNQ1OT1 Inhibition Combined with miR-370 Over-Expression Significantly Reduced Tumor Growth *In Vivo*

As shown in Figures 8A,B, knockdown of KCNQ1OT1 or over-expression of miR-370 reduced tumor growth. Further, knockdown of KCNQ1OT1 combined with over-expression of miR-370 exhibited the smallest tumor compared with each group in the experiment (*P* < 0.05). Similarly, the survival analysis demonstrated both KCNQ1OT1 inhibition and miR-370 restoration prolonged survival period compared with control group, and as expected, KCNQ1OT1 inhibition combined with miR-370 reintroduction contributed to the longest survival period (Figure 8C).

**Figure 8:** ***In Vivo* study. (A)** The stable expressing cells were used for the *in vivo* study. The nude mice carrying tumors from respective groups were shown. The sample tumor from respective group was shown. **(B)** Tumor volume was calculated every 4 days after injection, and the tumor was excised after 44 days. *P < 0.05 vs. Control group; ^#^*P* < 0.05 vs. pre-miR370 group; ^▲^*P* < 0.05 vs. sh-KCNQ1OT1 group. **(C)** The survival curves of nude mice injected into the right striatum (*n* = 15). *P* < 0.05 (pre-miR-370 or sh-KCNQ1OT1 group vs. Control group); *P* < 0.01 (pre-miR-370 + sh-KCNQ1OT1 group vs. Control group).

## Discussion

In this study, we demonstrated KCNQ1OT1 was up-regulated in glioma tissues and cells. Knockdown of KCNQ1OT1 suppressed the malignant behaviors of human glioma U87 and U251 cells. In addition, the KCNQ1OT1 knockdown up-regulated miR-370, which was lowly expressed in glioma tissues and cells. CCNE2 is a direct target of miR-370. We found that CCNE2 was up-regulated in glioma tissues. We further discovered that miR-370 played a tumor-suppressive role by down-regulating CCNE2 in glioma cells. The *in vivo* study demonstrated knockdown of KCNQ1OT1 combined with miR-370 over-expression produced the smallest tumor and the longest survival period in nude mice. Taken together, the KCNQ1OT1/miR-370/CCNE2 axis might exert an important role in human glioma tumorigenesis and malignant progression, which provided a novel promising therapeutic target.

The article "Knockdown of Long Non-Coding RNA KCNQ1OT1 Restrained Glioma Cells’ Malignancy by Activating miR-370/CCNE2 Axis" was retracted in 2023. Reason: concerns about the images.

Many research indicate that lncRNAs are abnormally expressed in multiple tumors, and play important roles in the biological processes of tumor cells (Bartonicek et al., 2016; Serghiou et al., 2016). LncRNA MALAT1 is up-regulated in pancreatic cancer, epigenetically inducing MALAT1 promotes tumor cell growth and invasion via regulating autophagy (Li et al., 2016). LncRNA TUG1 is highly expressed in hepatoblastoma tissues and cells, silencing TUG1 impairs cell proliferation, migration and invasion through increasing miR-34a-5p expression (Dong et al., 2016). KCNQ1OT1 encodes a paternally expressed long non-coding RNA, which has been shown to regulate the imprinting of several genes present at 11p15.5 locus in *cis* (Bliek et al., 2001; Higashimoto et al., 2006; Fedoriw et al., 2012; Schultz et al., 2015). KCNQ1OT1 aberrant expression is ubiquitous in various cancers. KCNQ1OT1 is up-regulated in Wilms’ tumor cells. Knockdown of KCNQ1OT1 promotes apoptosis of Wilms’ tumor cells (Yoshizawa et al., 2015). Consistent with previously reported, we proved that KCNQ1OT1 was highly expressed in glioma tissues and cells. Also, epigenetically silencing KCNQ1OT1 restrained proliferation, migration and invasion, while promoting apoptosis of glioma cells. Therefore, KCNQ1OT1 might be an oncogene in glioma and promote glioma cells’ malignant progression.

MiRNAs have various expression patterns and different biological functions in tumors. MiR-29a is highly expressed in breast cancer, and over-expressed miR-29a predicts shorter survival in patients with breast cancer. Inhibition of miR-29a impairs cell proliferation and weakens cell migratory abilities via up-regulating TET1 (Pei et al., 2016). MiR-497-5p exerts tumor-suppressive function in human angiosarcoma, reintroduction of miR-497-5p reduces KCa3.1 expression by targeting its mRNA 3′-UTR (Chen et al., 2016). MiR-370 is first identified as a tumor-suppressor in human cholangiocytes, and is found to be methylated by Interleukin-6 (Meng et al., 2008). MiR-370 exerts different function in various tumors. In most cases, miR-370 is lowly expressed and exerts tumor-suppressive role in tumor cells (Lo et al., 2012; Chen et al., 2014). A latest study shows that miR-370 is down-regulated in human glioma tissues cells (Peng et al., 2016). In addition, it has been confirmed that miR-370 inhibits glioma cells’ proliferation via targeting cyclin D1 and c-myc. Therefore, we further investigated the potential detailed function miR-370 might exert. As expected, our results showed that overexpression of miR-370 restrained glioma cells’ malignant progression, including cell proliferation, migration and invasion, while promoting apoptosis.

The article "Knockdown of Long Non-Coding RNA KCNQ1OT1 Restrained Glioma Cells’ Malignancy by Activating miR-370/CCNE2 Axis" was retracted in 2023. Reason: concerns about the images.

Recent studies have showed that lncRNAs can function as endogenous miRNA sponges by sponging miRNAs in a sequence-specific manner and impairing their function in a RISC manner. LncRNA NEAT1 promotes non-small cell lung cancer (NSCLC) cell via decreasing miR-377 expression. Mechanically, miR-377 targets NEAT1, and NEAT1 and miR-377 are in a RISC complex (Sun C. et al., 2016). Similarly, lncRNA MIR31HG harbors two miR-193b binding sites. MIR31HG and miR-193b respectively regulates each expression in a RISC manner (Yang et al., 2016). Our results showed KCNQ1OT1 exerted oncogenic role while miR-370 exerted the opposite function in glioma cells. Bioinformatics software (Starbase) indicated KCNQ1OT1 might harbor a binding site of miR-370. Luciferase reporter confirmed the binding site of miR-370 in KCNQ1OT1, and RIP assays supported the hypothesis that KCNQ1OT1 and miR-370 were in a RISC complex. Further, KCNQ1OT1 negatively regulated miR-370, and miR-370 inversely modulated KCNQ1OT1 expression. Knockdown of KCNQ1OT1 combined with miR-370 significantly restrained malignant behaviors of glioma cells *in vitro* and reduced tumor growth *in vivo*. Furthermore, KCNQ1OT1 inhibition combined with miR-370 over-expression significantly decreased CCNE2 and increased p-YAP expression. These results supported our assumption that KCNQ1OT1 promoted glioma cells progression via decreasing miR-370 expression. However, the underlying mechanism between miR-370 and CCNE2 remained unclear.

MiRNAs regulate cellular events by binding to the 3′-UTRs of downstream genes. For example, miR-208a-3p promotes gastric cancer cell proliferation via targeting PDCD4 3′-UTR (Yin et al., 2016). Meanwhile, miR-504 exerts tumor-suppressive function via targeting FOXP1 3′-UTR in glioma (Cui et al., 2016). In our study, three kinds of bioinformatics softwares indicated CCNE2 was a target of miR-370. Further, luciferase reporter results confirmed the binding site between miR-370 and CCNE2. CCNE2 belongs to the G(1) cyclin family and exerts important role in G1/S transition of the cell cycle (Payton and Coats, 2002). Dysregulation of CCNE2 has been reported in various tumors, such as breast cancer and NSCLC (Matsushita et al., 2015; Ye et al., 2016). In human prostate cancer, CCNE2 expression is elevated in tumor tissues (Wu et al., 2009, and when PTEN, which is conventionally lowly expressed in prostate cancer cells, is reintroduced, CCNE2 is blocked and results in cycle G(1) arrest (Macdonald et al., 2014). Moreover, miR-30a expression is negatively correlated with CCNE2 in prostate cancer pathological specimens (Zhang et al., 2016b). Similarly, CCNE2 expression is increased in NSCLC, over-expressed CCNE2 facilitates NSCLC cell growth and the effect can be abolished by reintroduction of miR-30d-5p (Chen et al., 2015). Consistent with previous studies, our results showed that CCNE2 expression was elevated in glioma tissues. Inhibition of CCNE2 hindered glioma cells progression. Also, CCNE2 inversed miR-370-induced suppression on glioma cells malignant behavior. Besides, a latest study shows CCNE2 is involved in regulation of Hippo pathway in breast cancer (Pegoraro et al., 2015). Hippo pathway is characterized as a tumor-suppressive axis, and plays important roles in tumor cellular process including proliferation, migration, invasion, and apoptosis (Alam et al., 2016; Atkins et al., 2016; Kemppainen et al., 2016; Mao et al., 2016). YAP is an important transcriptional activator and can be phosphorylated by Hippo pathway (Bouvier et al., 2016). Phosphorylation of YAP induces YAP functional nucleus localization transit to nonfunctional cytoplasmic cell distribution (LaQuaglia et al., 2016). We have demonstrated that KCNQ1OT1 regulated CCNE2 expression via decreasing miR-370 expression. Therefore, phosphorylated YAP expression were detected in cells treated with KCNQ1OT1 inhibition, miR-370 restoration and co-transfected KCNQ1OT1 inhibition and miR-370 restoration glioma cells. As expected, phosphorylated YAP expression was predominantly increased in cells co-transfected with KCNQ1OT1 inhibition and miR-370 restoration. This may partially declare the underlying mechanism of KCNQ1OT1/miR-370 regulation on glioma cells. The mechanism underlying tumorgenesis of human glioma cell lines by KCNQ1OT1 is schematically presented in Figure 9.

The article "Knockdown of Long Non-Coding RNA KCNQ1OT1 Restrained Glioma Cells’ Malignancy by Activating miR-370/CCNE2 Axis" was retracted in 2023. Reason: concerns about the images.

**Figure 9:** **The schematic cartoon of the mechanism of KCNQ1OT1 negatively regulated miR-370/CCNE2 axis in glioma**.

In conclusion, our study demonstrated that knockdown of KCNQ1OT1 inhibited glioma cells malignancy by up-regulating miR-370. Moreover, miR-370 suppressed glioma cells’ malignant biological behaviors by targeting CCNE2, and further activated Hippo pathway. Thus, therapy targeting KCNQ1OT1/miR-370/CCNE2 axis may be a promising option for the treatment of human gliomas.

## Author Contributions

YX contributed to the experiment design and implementation, manuscript draft and data analysis. JZ and WG contributed to the experiment implementation and data analysis. XL conceived or designed the experiments. JG, YG and WT performed the experiments. JC, ZL and JM analyzed the data. All authors read and approved the final manuscript.

## Conflict of Interest Statement

The authors declare that the research was conducted in the absence of any commercial or financial relationships that could be construed as a potential conflict of interest.
